The article "Scene Classification in the Environmental Art Design by Using the Lightweight Deep Learning Model under the Background of Big Data" was published in 2022. Journal: Comput Intell Neurosci.

# Scene Classification in the Environmental Art Design by Using the Lightweight Deep Learning Model under the Background of Big Data

**DOI:** 10.1155/2022/9066648

**Published:** 2022-06-13

**Authors:** Lu Liu

**Affiliations:** Department of Art and Design, Shaanxi Fashion Engineering University, Xi'an 710000, China

## Abstract

On the basis of scene visual understanding technology, the research aims to further improve the classification efficiency and classification accuracy of art design scenes. The lightweight deep learning (DL) model based on big data is used as the main method to achieve real-time detection and recognition of multiple targets and classification of the multilabel scene. This research introduces the related foundations of the DL network and the lightweight object detection involved. The data for a multilabel scene classifier are constructed and the design of the convolutional neural network (CNN) model is described. On public datasets, the effectiveness of the lightweight object detection algorithm is verified to ensure its feasibility in the classification of actual scenes. The simulation results indicate that compared with the YOLOv3-Tiny model, the improved IRDA-YOLOv3 model reduces the number of parameters by 56.2%, the amount of computation by 46.3%, and the forward computation time of the network by 0.2 ms. It means that the IRDA-YOLOv3 network obtained after the improvement can realize the lightweight of the network. In the scene classification of complex traffic roads, the classification model of the multilabel scene can predict all kinds of semantic information of a single image and the classification accuracy for the four scenes is more than 90%. In summary, the discussed classification method based on the lightweight DL model is suitable for complex practical scenes. The constructed lightweight network improves the representational ability of the network and has certain research value for scene classification problems.

## 1. Introduction

The environmental art design is an artistic activity that comprehensively utilizes various artistic means and engineering techniques to create a scientific living environment for people [1]. The purpose of the environmental art design is to increase the beauty of the scene space through systematic art design while continuously meeting the functional needs of human beings. Whether it is interior design or exterior design, it is the goal of the environmental art design to strive to make the space environment have a beautiful sense of the times. The concept of modern environmental art design calls for returning to nature and pursuing simplicity and fashion [2, 3]. With ecological balance as the core, human activities are integrated into the objective laws of nature, to realize the humanization of nature and the naturalization of human beings. It is neither the solipsistic mentality of conquering nature and looking down on everything, nor the fear and compromise of natural forces but the true unity of man and nature.

Using the combination of emerging scientific and technological achievements and historical culture to meet the aesthetic pursuit of human beings in the new era is the new requirement of aesthetic design in environmental art design. Environmental art design delights body and mind, beautifies life, and improves the sustainability of life through the aesthetic characteristics of design works. It is the role of design aesthetics in the application of environmental art design [4–6]. Among the computer technologies that integrate art and design, scene visual understanding is the most widely used technology. In the current era of big data, the application of deep learning (DL) technology in various visual tasks and the analysis of massive data have a certain role in promoting. In the problem of environmental art scene classification, it needs to be based on object detection. Since object detection based on handcrafted features is easily affected by the quality of feature selection. Therefore, it is easy to cause poor application effects in actual scenarios. Using the feature extraction method based on DL, the convolutional neural network (CNN) can be used to extract deeper features, which has the advantages of high detection accuracy and automatic feature extraction [7–9].

Considering the scene classification problem in environmental art design, it is of great significance for multilabel scene analysis and subsequent intelligent decision-making in real life. Since CNN can be used for model training through massive data, in the scene classification, the lightweight DL model based on big data is used as the main method to realize the real-time detection and recognition of multiple targets and the classification of multilabel scenes. Firstly, the involved DL network and the relevant basics of lightweight object detection are introduced; secondly, the data of the multilabel scene classifier is constructed, and the design of the CNN model is described. Finally, the effectiveness of the lightweight object detection algorithm is verified on public datasets to ensure its feasibility in practical scene classification. The innovation lies in the improvements to the YOLOv3-Tiny network. A lightweight network architecture IRDA-YOLOv3 with a stable detection effect and small computing requirement is proposed, which improves the representational ability of the network and can more effectively solve the problem of scene classification.

## 2. Materials and Methods

### 2.1. Scene Visual Understanding in Environmental Art Design

With the gradual development of society, politics, economy, and culture, the relationship between environmental design and human beings has become closer. It transforms the environment of people's production, life, work, and study by means of technology and art to create a place suitable for various needs of human beings and to achieve a beautiful environment that meets people's spiritual and material needs [10]. The direct purpose of the environmental art design is to make the space atmosphere harmonious and orderly while expressing the design concept. Environmental design uses certain organization and enclosure methods to artistically process the space interface and uses natural light, artificial lighting, furniture, decorations, layout, modeling, and other design languages, as well as the configuration of plants and flowers, water bodies, sculptures, etc. [11–13]. The indoor and outdoor space environment of the building reflects a specific atmosphere and a certain style to meet people's functional use and visual aesthetic needs.

In complex scenes and images of the environmental art design, there are usually situations such as occlusion of target objects, different shapes, and changes in color difference. These factors directly affect the feature extraction effect of target information [14]. Therefore, the application of scene visual understanding algorithm in art-aided design plays an important role in extracting scene information and outputting clear images. The main design process is shown in Figure 1. In the process of art-aided design, first, the color of the scene image should be segmented based on the set threshold; next, a series of morphological processing is performed on the effective description area to obtain the candidate region; finally, the local feature extraction is performed. The relevant algorithm is used to obtain the features of the candidate region, and the combination design is carried out according to the feature results.

In scene understanding, image segmentation plays a crucial role as a preprocessing step of the algorithm. The specific scene image segmentation algorithm is shown in the following equation:

(1) $$\begin{array}{c} \left(x,y\right)=f_{1}\left(x,y\right),\\ f_{2}\left(x,y\right). \end{array}$$

Here, *x*, *y* refers to the horizontal and vertical coordinates of the plane where the image is located. Through *f*_1_(*x*, *y*) can achieve the effect of effectively eliminating the interference of the blue area in the image, and by introducing *f*_2_(*x*, *y*), the interference of colors with a large color difference with blue, such as black, red, and green can be eliminated.

After the color segmentation of the image is completed, a series of morphological processing needs to be performed on the regions that effectively describe the shape in the image, to reduce or avoid the influence of noise as much as possible. *A* and *B* are set to be a set in two-dimensional space, and the fractured parts of some candidate regions are recleaved through the expansion operation. *B* dilation *A* is defined as the set of all *Z* displacements. To make sure that there is at least one overlapping element in *A* and *B*, and then the morphological operation is performed, which includes corrosion expansion operations, contour smoothing operations, and breaking narrow gaps. To reduce the influence of interference on the effect of acquiring candidate scene regions, it is necessary to clarify the rules for extracting candidate scene regions. The connected area is set as *C*_*i*_ (where *i* refers to the first connected area). *L*_*i*_, *W*_*i,*_ and *S*_*i*_ represent the width, height, and area of the connected area, respectively. When the three meet the conditions of equations (2) to (4), it means that the connected area is a candidate region.

(2) $$\begin{array}{c} S_{i}\geq S_{\min}\cap S_{i}\leq S_{\max}, \end{array}$$

(3) $$\begin{array}{c} \frac{L_{i}}{W_{i}}\geq {\left(\frac{L}{W}\right)}_{\min}\cap L_{i}/W_{i}\leq {\left(\frac{L}{W}\right)}_{\max}, \end{array}$$

(4) $$\begin{array}{c} \frac{S_{i}}{L_{i}}\times W_{i}\geq {\left(\frac{S}{L}\times W\right)}_{\min}. \end{array}$$

Here, *S*_min_ and *S*_max_ express the minimum and maximum value of the area of the connected area, respectively; (*L*/*W*)_min_ and (*L*/*W*)_max_ refer to the minimum and maximum value of the aspect ratio, respectively.

To complete the extraction of target features inside the scene in a more detailed manner, the gradient and direction of each pixel in the 16 × 16 window range are usually calculated with the Scale Invariant Feature Transform (SIFT) feature point as the center in the candidate region. SIFT features not only have scale invariance, even if the rotation angle, image brightness, or shooting angle of view are changed, but good detection results can also still be obtained [15–17]. The SIFT algorithm takes the detected key points as the center, selects a 16 × 16 neighborhood, and then divides the neighborhood into 4 *∗* 4 subregions. Then, the gradient direction is divided into 8 intervals, so that a 4 × 4 × 8 = 128-dimensional feature vector will be obtained in each subarea. It is proposed that the eigenvectors of the neighborhood should be normalized after the eigenvectors are obtained, and the normalization direction is the main direction of calculating the neighborhood key points. The neighborhood is rotated to a specific direction according to the principal direction, which makes the feature rotation-invariant. Then, according to the size of each pixel in the neighborhood, the neighborhood is scaled to the specified scale, which further makes the feature description scale-invariant. The core idea of the SIFT algorithm is shown in Figure 2.

The SIFT algorithm can be decomposed into the following four steps: (1) detection of extremum in scale-space: search for image locations on all scales. The potential scale and rotation invariant points of interest are identified by a Gaussian differential function. (2) Localization of key points: at each candidate location, the location and scale are determined by a well-fitted model. The selection of key points is based on the degree of stability. (3) Determination of the direction: based on the local gradient direction of the image, one or more directions are assigned to each key point position. All subsequent operations on image data are transformed relative to the orientation, scale, and position of key points, thereby providing invariance to these transformations. (4) Description of key points: in the neighborhood around each key point, the local gradient of the image is measured at the selected scale. These gradients are transformed into a representation that allows for relatively large local shape deformations and lighting changes.

### 2.2. Scene Description and Target Detection Based on DL under Big Data

In the context of big data, raw video is a kind of unstructured data, the content of which cannot be directly understood by the computer and reflects the relevant content [18]. The structured description of the scene mainly includes three levels, which are the description of the essence of the object, the description of the attributes of the object, and the description of the attribute relationship between the objects. It has become the latest technological progress to extract high-level semantic features with DL, so as to structure the description of video scenes. The structured description model of scene video is essentially a rich semantic model, which is used to parse the content of video events until intuitive text information is obtained [19–21]. It can describe the semantics of video events and save them into text information, so that it can be understood by humans and computers.

A Video Structurized Description (VSD) model is proposed, and its framework is shown in Figure 3. The video streaming of the scene is used as the input information of the input terminal, which mainly refers to the video semantic content including objects, attributes, and features, including low-level semantics and high-level semantics [22, 23]. The VSD model framework includes three parts: basic module, content analysis module, and application module, and its general structure is shown in Figure 3. These three parts are combined with ontology knowledge and reasoning logic to construct the basis of VSD. Among them, the focus of the semantic module is the structured class of the video ontology, and the partial data obtained after the preprocessing of the video is used as the input information of the input terminal of the module, and then a structured description ontology of the video event is formed. The structure of video can be regarded as a semantic web, which is essentially a nonrelational data set. The specific structured classes mainly include objects, events, activity networks, spatial relationships, and motion states. The use of these structured classes to generate event ontology is the key link in the process of VSD [24–26]. After the event ontology instance is created, the content analysis module needs to complete the reasoning of the ontology data. The basis for realizing event description lies in object semantics, so it is necessary to transform semantics into textual information that can be understood by humans through the basis of objects and related descriptions. The final application module is mainly responsible for fully realizing and applying the information inferred from the model in the upper-layer application. The application module can convert the input video streaming into the output of related events by adjusting the application interface of video structured description.

Object recognition in VSD is very critical. Since the operation of traditional object detection and recognition methods requires the extraction of many different features, DL technology has become the current research focus in the field of computer vision. For the CNN in DL, its basic structure mainly includes two modules: feature extraction and feature mapping [27–30]. In the part of feature extraction, the input of each layer of nodes and the upper local receptive field are correlated with each other, to obtain the corresponding features and clarify the positional relationship between the features. In the part of feature mapping, the computation in the neural network (NN) can be regarded as being composed of multiple feature maps and all nodes have the same weights [31, 32]. Considering the hardware equipment of the experiment, the designed network structure is composed of two convolutional layers, two pooling layers, and two fully connected layers. The size of the convolution kernel is 5 × 5, and the network structure is shown in Figure 4. The ReLU function is selected as the activation function of the convolutional layer, the data set is divided into training set and test set, and the mean value is processed in the data preprocessing link.

Because CNN needs a large number of samples, when the positive samples are set to be *B* Bounding Boxes, the effect is very poor. To further improve the accuracy of positioning, RCNN performs Bounding Box regression after nonmaximum suppression (NMS) and further fine-tuning the location of the Bounding Box. Unlike the Bounding Box regression of the Deformable Parts Model (DPM), RCNN is a regression performed at the Pool5 layer. The Bounding Box is category-related, that is, the parameters of the Bounding Box regression of different categories are diverse.

### 2.3. Scene Classification Algorithm Based on Lightweight DL

Network lightweight is talking about using fewer network parameters to meet or exceed the performance of existing CNN. At present, many target detection and classification based on CNN have problems of low storage, low energy consumption, and low computing power. Due to resource constraints, the model is difficult to implement in terms of deployment and usage. Therefore, in the task of target detection, the NN needs to be light-weighted to better realize the feature extraction task of the detector. Among the regression-based target detection algorithms, the YOLO-Tiny series of lightweight detection algorithms are proposed for embedded devices [33–35]. Similar to the YOLO series of algorithms, the classification problem in images needs to be transformed into a regression problem first. The specific operation is to divide the input image into *S* × *S* grids, each grid generates a Bounding Box according to the prior information and predicts and outputs 4 position information for each Bounding Box, as well as the category of the predicted Bounding Box.

YOLOv3-Tiny removes some feature layers on the basis of YOLOv3 and only retains 2 independent prediction branches. YOLOv3-Tiny is a multitask, end-to-end, attention mechanism, and multiscale. Multitask is to complete the classification and regression of the target at the same time, realize parameter sharing, and avoid overfitting. End-to-end means that the model directly gives the prediction information of classification and regression after receiving the image data. The attention mechanism is to focus on the features of the target region for detailed processing and to improve the processing speed. The feature of multiscale is to fuse downsampling and upsampling data with each other, and its function is to segment objects of various scales.

When training the model, methods such as Mosaic data augmentation, label smoothing, and cosine annealing with learning rate decay can be used to improve the training speed and detection accuracy of the model. Since the same target will predict multiple candidate Bounding Boxes, the NMS method is used to suppress redundant candidate regions, and the final predicted Bounding Box is output. The network structure of YOLOv3-Tiny is shown in Figure 5. Three residual units are used, Leaky ReLU is used as the activation function, two feature layers are used for the classification and regression of the target, and the Feature Pyramid Network (FPN) is used when merging the effective feature layers. It also uses the CSPNet structure and performs channel segmentation on the feature extraction network. The feature layer channel output after 3 × 3 convolutions is divided into two parts, and the second part is taken.

To ensure that the accuracy and real-time performance of the model are in a balanced state when dealing with object detection problems, the YOLOv3-Tiny network is improved. A lightweight network architecture IRDA-YOLOv3 with a stable detection effect and small computing power requirement is proposed. The network uses a multilayer feature map fusion algorithm for feature fusion, makes full use of multilayer shallow network features to improve the accuracy of target detection, and uses point convolution to increase the depth of the network structure. When designing a lightweight network structure, the original part of the convolutional layer is retained as much as possible, and the increase in the number of convolutional layers is avoided. Using the weight feature in the attention mechanism of the IRDA module, the spatial features of the deep network are recalibrated, so that the network can learn more useful feature information before the output layer features and improve the final classification effect.

The Pytorch DL framework is used to build independent data loading methods for each category. Meanwhile, to solve the problem of unbalanced samples, the weight processing method of weighted cross entropy loss is adopted. The cross-entropy loss function can be expressed as follows:

(5) $$\begin{array}{c} L=-\sum_{i}t_{i}*\;\log\;y_{i}, \end{array}$$

where *y*_*i*_ is the output value of the NN, and *t*_*i*_ is the correct label value.

When using weighted cross-entropy loss, its equation is shown as follows:

(6) $$\begin{array}{c} L=-\sum_{i}a*t_{i}*\;\log\;y_{i}, \end{array}$$

(7) $$\begin{array}{c} \left\{\begin{array}{cc} a>1, & \text{if }i=k,\\ a=1, & \text{if }i\neq k, \end{array}\right. \end{array}$$

where *a* is the weight parameter, when the category is *k* class, the weight value of *a* is greater than 1, and when the category is not *k* class, the weight value of *a* is equal to 1.

### 2.4. Design of Simulation Experiment

The performance of the improved lightweight target pretest algorithm is mainly verified on the International Open Autonomous Driving Database (KITTI). The KITTI dataset was cofounded by the Karlsruhe Institute of Technology in Germany and Toyota American Institute of Technology. It is currently the largest evaluation dataset of computer vision algorithms in the world for autonomous driving scenarios. The hardware equipment of the relevant experiments is GeForce GTX TITAN X, the graphics chip is Intel Core i7 CPU@3,40 GHz 3.40 GHz, the system is Ubuntu16.04, the programming language is Python, the training framework is Pytorch, and the DL framework is tensorflow1.12.0. The training batch of the model is set to 32, the learning rate is 0.001, the weight decay factor is 0.0005, and the maximum number of iterations is 60000.

On the VOC2007 test data, the performance of several lightweight YOLO series models is compared and analyzed. The evaluation indicators include model scale, forward inference time, and mAP.

Several networks such as SqueezeNet, YOLOv-Tiny, and YOLOv3-Tiny are selected as controls to evaluate the performance of the improved IRDA-YOLOv3 lightweight detection algorithm. Evaluation indicators include structural parameters (Params), moving average confluence statistics (MACS), and inference speed (Speed).

## 3. Results and Discussion

### 3.1. Performance Comparison of Different Networks in YOLO Detection Algorithm

The performance of different networks in the YOLO detection algorithm is compared, and the results are shown in Figures 6 and 7. Among them, Params represents the weight parameters of all parameterized layers of the model in the network; MACS expresses the number of fixed-point multiply-accumulate operations performed per second; Speed refers to the forward inference time of the network processing an image when the input image is input. In the process of improving the model, the feature layer of the high-dimensional channel is recalibrated with dimension features mainly for the part near the output layer at the back end of the network. According to the results in the figure, it demotes that although SqueezeNet has advantages in Params and MACS, which is slightly higher than YOLOv3-Tiny, its Speed indicator is lower than IRDA-YOLOv3. The calculation shows that compared with the YOLOv3-Tiny model, the improved IRDA-YOLOv3 model reduces the number of parameters by 56.2%, the amount of computation by 46.3%, and the forward computation time of the network by 0.2 ms. It means that the improved IRDA-YOLOv3 network can achieve network lightweight.

### 3.2. Multitarget Detection Performance of Lightweight DL Networks

Based on the above-given experimental results, several lightweight models are compared with the IRDA-YOLOv3 model and the performance is evaluated in terms of the model scale, forward inference time, and mAP. The specific results are shown in Figures 8 and 9. The experimental results indicate that the constructed IRDA-YOLOv3 model incorporates the inverse residual depth, so its performance is better than that of YOLOv3-Tiny, with a 56.0% reduction in size and parameter performance and a 3.9 mAP improvement in detection accuracy.

To more intuitively compare the improvement in detection accuracy performance of IRDA-YOLOv3, the performance of YOLOv3-Tiny and IRDA-YOLOv3 are compared in different categories of the test set. The comparison results of the average accuracies of the two algorithms on the test set in the car and pedestrian databases are shown in Figure 10.

### 3.3. Performance Evaluation of Scene Classification

In the complex traffic road scene classification, it is very important to extract effective road scene information from a single image and train an efficient classification model to understand the real complex scene. The multilabel scene classification model based on the multibranch task approach achieves the best performance of the model on the 56th Epoch. In the test set, the comparison of the correct rate of scene classification for four categories is evaluated, and the results are shown in Figure 11. It demonstrates that the multilabel scene classification model can predict various semantic information of a single image. In practical applications, it can help the system to determine whether the current road scene will affect the visual warning.

## 4. Conclusions

Structural description of scenes in environmental art design is a comprehensive problem. For detecting objects in a video scene, it is necessary to organize the relationship between objects through an appropriate logical language. The input image is taken as a feature and extracts low-dimensional features that can generalize the image statistics or semantics. The purpose of this class of methods is to improve the robustness of scene classification. The traditional artificial design features are mostly based on the underlying semantic feature information of the image, so it is difficult to describe the high-level semantic information of the image. The CNN in DL is used to complete feature extraction, and the learned features have strong generalization performance.

To ensure that the accuracy and real-time performance of the model are in a balanced state when dealing with object detection problems, the YOLOv3-Tiny network is improved. A lightweight network architecture IRDA-YOLOv3 with a stable detection effect and small computing power requirement is proposed. The network uses a multilayer feature map fusion algorithm for feature fusion, makes full use of multilayer shallow network features to improve the accuracy of target detection, and uses point convolution to increase the depth of the network structure. The constructed IRDA-YOLOv3 model incorporates the inverse residual depth, so its performance is better than that of YOLOv3-Tiny, with a 56.0% reduction in size and parameter performance, and a 3.9 mAP improvement in detection accuracy. In the scene classification of complex traffic roads, the classification model of the multilabel scene can predict all kinds of semantic information of a single image, and the classification accuracy for the four scenes is more than 90%. The constructed lightweight network integrates contextual feature information, improves the representation ability of the network, and has a certain value for solving scene classification problems. However, there is no in-depth discussion on how to further optimize CNN. Therefore, it is still a significant direction to improve the performance and stability of the algorithm in the followup research.

## Figures and Tables

**Figure 1:** Art-aided design process incorporating a visual understanding of the scene.

**Figure 2:** The core idea of the SIFT algorithm.

**Figure 3:** Rough framework of the VSD model.

**Figure 4:** The network structure of CNN.

**Figure 5:** The network structure of YOLOv3-tiny.

**Figure 6:** Parameter calculation comparison of different networks.

**Figure 7:** Comparison of the speed of different networks.

**Figure 8:** Comparison of scale and forward inference time for different lightweight models.

**Figure 9:** mAP performance comparison of different lightweight models.

**Figure 10:** The comparison of the average accuracies of the two algorithms on the test set in the car and pedestrian databases.

**Figure 11:** The accuracy of the optimal iterative model for scene classification in 4 categories.

## Data Availability

The data used to support the findings of this study are included within the article.
